# Evaluation of Traumatic Subdural Hematoma Volume by Using Image Segmentation Assessment Based on Deep Learning

**DOI:** 10.1155/2022/3830245

**Published:** 2022-06-28

**Authors:** Dan Chen, Lin Bian, Hao-Yuan He, Ya-Dong Li, Chao Ma, Lian-Gang Mao

**Affiliations:** ^1^Department of Neurosurgery, The Third People's Hospital of Hefei, Hefei 230022, China; ^2^Department of Neurosurgery, HwaMei Hospital, University of Chinese Academy of Sciences, Ningbo Institute of Life and Health Industry, University of Chinese Academy of Sciences, Ningbo 315010, China; ^3^Department of Clinical Laboratory, HwaMei Hospital, University of Chinese Academy of Sciences, Ningbo 315010, China

## Abstract

Rapid and accurate evaluations of hematoma volume can guide the treatment of traumatic subdural hematoma. We aim to explore the consistency between the measurement results of traumatic subdural hematoma (TSDH) using a deep learn-based image segmentation algorithm. A retrospective study was conducted on 90 CT images of patients diagnosed with TSDH in our hospital from January 2019 to January 2022. All image data were measured by manual segmentation, convolutional neural networks (CNN) algorithm segmentation, and *ABC*/2 volume formula. With manual segmentation as the “golden standard,” a consistency test was carried out with CNN algorithm segmentation and *ABC*/2 volume formula, respectively. The percentage error of CNN algorithm segmentation is less than *ABC*/2 volume formula. There is no significant difference between CNN algorithm segmentation and manual segmentation (*P* > 0.05). The area under curve of the *ABC*/2 volume formula, manual segmentation, and CNN algorithm segmentation is 0.811 (95% CI: 0.717~0.905), 0.840 (95% CI: 0.753~0.928), and 0.832 (95% CI: 0.742~0.922), respectively. From our results, the algorithm based on CNN has a good efficiency in segmentation and accurate calculation of TSDH hematoma volume.

## 1. Introduction

Traumatic subdural hematoma (TSDH) is a common disease in neurosurgery [1]. The pathogenesis of this disease is mainly that the patient's head is violently hit, which causes the dura mater of his brain tissue to shift. Eventually, the bridging vein between the cerebral cortex and venous sinus was broken, which led to bleeding [2, 3]. At present, patients with this disease are mainly clinically treated by surgery or conservative treatment [4, 5]. After the onset of TSDH, patients will have symptoms such as increased intracranial pressure, coma, cerebral hernia, and hemiplegia. Some patients will have dilated pupils, a severe threat to their physical and mental health and life safety [6]. Therefore, accurate calculation of hematoma volume for patients has important guiding significance for later treatment and prognosis.

Previous studies have found that for TSDH, drainage of only 20% of hemorrhage can effectively help hematoma absorption [7]. There are many methods for measuring and calculating different types of intracranial hemorrhage. The traditional manual segmentation method is the “gold standard” for calculating hematoma volume, but it is time-consuming and laborious [8, 9]. Another conventional method is Tada formula, namely, *A* × *B* × *C*/2 volume formula [10]. Although this method is suitable for subdural hematoma, the shape of subdural hematoma is not all symmetrical crescent, especially since many chronic subdural hematomas are comma-like [11]. The accuracy of the calculation results is controversial [12, 13].

With the development of computer technology such as deep learning, more and more scholars began to try to calculate the hematoma volume by using related technologies [14–16]. Yu et al. [17] constructed a deep learning algorithm covering all types of intracerebral hemorrhage hematoma volume. This algorithm has high accuracy and consistency with manual segmentation estimation of cerebral parenchymal hemorrhage hematoma volume. However, there is no specific algorithm for subdural hematoma at present. This study is aimed at proposing a segmentation method based on the CNN algorithm and compare it with Tada formula and manual segmentation to explore an accurate and convenient measurement method for subdural hematoma volume.

## 2. Methods

### 2.1. General Information

A total of 90 patients with TSDH diagnosed by CT in our hospital from January 2019 to January 2022 were collected retrospectively. There were 67 males and 23 females, aged from 23 to 80 years, with an average of (56.5 ± 13.9) years.

Inclusion criteria are (1) select CT images of the head of patients with subdural hematoma. (2) All of them were obtained before or without surgery. (3) All of them are in standard DICOM format, and the scanning parameters and machine brands are not limited. (4) Age > 18 years old. Exclusion criteria were patients with bilateral subdural hematoma.

### 2.2. Manual Segmentation

DICOM-formatted CT scan images of each patient were imported into Insight Toolkit SNAP open source software. Using manual segmentation, two radiologists manually sketched a three-dimensional region of interest (ROI) layer by layer along the hematoma boundary on the cross-sectional CT plain scan image and output the hematoma volume.

### 2.3. Tada Volume Formula

Tada volume formula measurement regards cerebral hemorrhage focus as an ellipsoid. A physician calculated the blood loss with 3 years of experiences in neuroimaging diagnosis. The specific calculation formula is

(1) $$\begin{array}{c} V\left(\text{bleeding}\right)=A\times B\times C\times \frac{1}{2}. \end{array}$$

Tada volume formula can be expressed by *ABC*/2 volume formula [18]. The detailed calculation process is that *A* is the largest length (anterior to posterior) of the SDH, *B* is the maximum width (lateral to midline) 90° to *A*, and *C* is the maximum height (coronal plane or multiplication of slices) of the hematoma.

### 2.4. Deep Learning Segmentation

#### 2.4.1. Construction Model

The Deep Red AI Toolbox generates the deep learning model in this research. To reduce the overfitting risk of the segmentation result of the construction algorithm and improve the robustness, the CT images of the included cases were verified by 5-fole crossover method [19]. According to the ratio of training set to test set of 4 : 1, 90 patients were divided into training set (*n* = 72) and test set (*n* = 18). Four groups were selected as the training set, the remaining one group was selected as the verification set, and five training times were conducted. Summarize the results of five models in their respective verification sets to evaluate the performance of algorithm models (Figure 1).

#### 2.4.2. Radiomics Feature Extraction

The convolutional neural network (CNN) has good feature extraction performance, so this paper chooses a convolutional neural network to extract image features to get the best image fusion result. Firstly, the CT image is preprocessed by fusion, and the hematoma area on the image is automatically detected and segmented by CNN algorithm (Figure 2). The software automatically measures the bleeding volume and records the measurement results.

The image is deaveraged when the CNN algorithm analyzes the image, as shown in the following formula.

(2) $$\begin{array}{c} a^{*}=a-\lambda . \end{array}$$

The *λ* is the mean value of the image set. *a* is the characteristic value.

A complete CNN is a multilayer structure, including input layer, pooling layer, full connection layer, and convolution layer. Convolution layer is the most critical part, which contains many neural network nodes and can extract the features of image fusion. The operation of convolution layer can be described as the following formula.

(3) $$\begin{array}{c} a_{j}^{l}==e\;\left(\underset{i}{\sum }\in N_{j}a_{j}^{l-1}\times h_{ij}^{l}+d_{j}^{l}\right). \end{array}$$

Because of the large number of image features, it is necessary to reduce the dimension of image fusion features. This step is mainly realized through the pooling layer, and the optimal image fusion features are identified through the maximum pooling function, which can be described as the following formula.

(4) $$\begin{array}{c} a_{j}^{l}=\text{down}\left(a_{j}^{l-1}\right). \end{array}$$

*l* represents the number of feature layers. *a*_*j*_^*l*−1^ represents the jth feature of the *l* − 1 layer.

In the training process, the segmentation accuracy on the loss function and verification set is checked in real time, the convergence speed and trend are judged, and the network parameters are adjusted. Satisfactory model is obtained in training set, and algorithm segmentation result is obtained in test set.

### 2.5. Measurement Error of Segmentation Method

The CT image data included in this study used manual image segmentation method, *ABC*/2 volume formula measurement method, and the CNN algorithm image segmentation method to measure hematoma volume. The results measured by CT manual segmentation method are “gold standard” [20]. The specific process is shown in Figure 3. In addition, the absolute percentage error (APE) is used to represent the measurement error, and the specific calculation formula is

(5) $$\begin{array}{c} \text{APE}=\frac{\left|V_{m}-V_{r}\right|}{V_{r}}\times 100\%. \end{array}$$

*V*_*m*_ and *V*_*r*_ represent the measured and actual value of bleeding volume, respectively.

### 2.6. Statistical Analysis

SPSS 23.0 statistical software was used for data processing and analysis. Measurement data is expressed by mean ± standard deviation. Group comparison was performed by independent sample *t* test. Measurement data with nonnormal distribution are expressed by median and quartile interval [*M* (*P*_25_, *P*_75_)], and the Mann–Whitney *U* test is used. *P* ≤ 0.05 indicates that the difference is statistically significant.

## 3. Results

### 3.1. Volume of Subdural Hematoma Measured by Different Image Segmentation Methods

After examination and calculation, the percentage error of hematoma volume obtained by the CNN algorithm segmentation, *ABC*/2 volume formula segmentation, and the manual segmentation is shown in Table 1. Taking the manual segmentation result as the “golden standard,” the percentage error of CNN algorithm segmentation is less than *ABC*/2 volume formula. In addition, there was significant difference between *ABC*/2 volume formula segmentation and manual segmentation (*P* > 0.05). However, there was no significant difference between CNN algorithm segmentation and manual segmentation (*P* < 0.05) (Figure 4).

### 3.2. Evaluation of Model Prediction Efficiency

The area under curve (AUC) of the *ABC*/2 volume formula is 0.811 (95% CI: 0.717~0.905). The AUC of the manual segmentation is 0.840 (95% CI: 0.753~0.928). The AUC of the CNN algorithm segmentation is 0.832 (95% CI: 0.742~0.922). It is suggested that the segmentation result of CNN algorithm is closer to the manual segmentation than the *ABC*/2 volume formula (Figure 5).

## 4. Discussion

TSDH is one of the common secondary injuries of traumatic brain injury, accounting for about 40% of traumatic intracranial hematoma. It is still one of the main causes of traumatic brain injury death [21]. With the increase of traffic accidents and falling accidents, the incidence of this disease is increasing year by year [1]. The brain function of patients with TSDH is seriously damaged, and there are many kinds of dysfunction, which is a serious threat to patients' health and life safety [22]. Therefore, it is of great significance to make a clear diagnosis of the disease and determine the exact volume of hematoma to guide clinical treatment.

The calculation method of Tada formula is simplified from the ellipsoid volume formula, which is widely used in the measurement of cerebral parenchymal hemorrhage and hematoma as a simple and fast estimation tool for hematoma volume beside the bed [23, 24]. Previous studies have shown that the correlation between *ABC*/2 volume formula and manual segmentation algorithm in acute subdural hematoma is high, but lower than parenchymal hemorrhage [25]. However, the percentage error of Tada formula in our study was larger than that in previous studies. The reason may be that the error of Tada formula increased with the increase of hematoma volume.

In order to make up for the deficiency of traditional algorithms, more and more researches have applied CNN correlation algorithms for hematoma segmentation in recent years [14, 19]. In this study, an automatic segmentation algorithm of intracranial hematoma based on CNN is adopted, automatically identifying and segment subdural hematoma displayed by head CT plain scan and calculating the hematoma volume. Taking the manual segmentation method as the “gold standard” [26], the consistency of CNN algorithm segmentation and *ABC*/2 volume formula is tested, respectively. The results show that the percentage error of CNN algorithm segmentation is less than *ABC*/2 volume formula. This shows that the hematoma volume segmented by CNN algorithm is closer to manual segmentation. In addition, there was no significant difference between CNN algorithm segmentation and manual segmentation. However, in this study, the 5-fold crossover test was adopted, and the data set was randomly divided into five groups in turn as the training set and test set. The final results showed the average capability of the models [20].

To better grasp the disease condition and answer clinical questions more accurately, especially for the inaccurate calculation of subdural hematoma by traditional multifield formula, it is a challenge faced by clinicians. In addition, there is a big error in the multifield formula, and manual segmentation is time-consuming and laborious, limiting its application in the study of the relationship between hematoma volume and prognosis [27]. With the in-depth application of artificial intelligence technology in clinical medicine, it is possible to accurately and conveniently segment intracranial hematoma and explore hematoma volume as an indication of operation [28]. In our study, the AUC of the CNN algorithm segmentation is 0.832 (95% CI: 0.742~0.922). At the same time, that of the manual segmentation is 0.840 (95% CI: 0.753~0.928). It shows that the CNN algorithm segmentation method is closer to the manual segmentation method. More algorithms can be applied to evaluate the subdural hematoma in the future [29].

## 5. Conclusions

In the TSDH patients, compared with the traditional *ABC*/2 volume formula, the CNN algorithm used to calculate the volume of hematoma in head CT plain scan images is in good agreement with the manual segmentation results. However, the cases included in this study were single centers, and the sample size was small. There was some error in the algorithm segmentation. Therefore, the clinical application needs further exploration.

## Figures and Tables

**Figure 1:** Convolution neural network modeling flow chart.

**Figure 2:** Region of interest intercepted by convolutional neural network model. (a) Origin image. (b) Image clipping. (c) Extraction of eigenvalues of the ROI. (d) Extracted hematoma.

**Figure 3:** Image segmentation flow chart.

**Figure 4:** Comparison of the mean value of hematoma volume among three image segmentation methods. ∗*P* < 0.05.

**Figure 5:** Receiver operating characteristic curve analysis of different segmentation methods.

**Table 1:** Volume and percentage error of subdural hematoma measured by different image segmentation methods [*M* (*P*_25_, *P*_75_)] (ml).

Methods	Volume	Minimum	Maximum	Percentage error (%)
Manual segmentation	26.15	7.43	44.46	—
CNN segmentation	21.38	4.31	38.44	19.48 (11.45, 52.43)
*ABC*/2 volume formula	38.90	13.52	63.64	24.53 (14.25, 43.85)

Note: “-”: not available.

## Data Availability

The data used to support the findings of this study are available from the corresponding author upon request.
